# A new modification of the flexible Weibull distribution based on power transformation: Monte Carlo simulation and applications

**DOI:** 10.1016/j.heliyon.2023.e17238

**Published:** 2023-06-16

**Authors:** Faridoon Khan, Zubair Ahmad, Saima K. Khosa, Mohammed Ahmed Alomair, Abdullah Mohammed Alomair, Abdulaziz khalid Alsharidi

**Affiliations:** a Pakistan Institute of Development Economics, Islamabad 44000, Pakistan; b Department of Statistics, Quaid-e-Azam University, Islamabad 44000, Pakistan; c Department of Mathematics and Statistics University of Saskatchewan, Saskatoon, SK, Canada; d Department of Quantitative Methods, School of Business, King Faisal University, Al-Ahsa 31982, Saudi Arabia; e Department of Mathematics and Statistics, College of Science, King Faisal University, Al Ahsa 31982, Saudi Arabia

**Keywords:** Weibull distribution, Flexible Weibull distribution, Beta power transformation, Estimation, Simulation, Failure times data, Statistical modeling

## Abstract

Statistical modeling is a crucial phase for decision-making and predicting future events. Data arising from engineering-related fields have most often complex structures whose failure rate possesses mixed state behaviors (i.e., non-monotonic shapes). For the data sets whose failure rates are in the mixed state, the utilization of the traditional probability models is not a suitable choice. Therefore, searching for more flexible probability models that are capable of adequately describing the mixed state failure data sets is an interesting research topic for researchers. In this paper, we propose and study a new statistical model to achieve the above goal. The proposed model is called a new beta power very flexible Weibull distribution and is capable of capturing five different patterns of the failure rate such as uni-modal, decreasing-increasing-decreasing, bathtub, decreasing, increasing-decreasing-increasing shapes. The estimators of the new beta power very flexible Weibull distribution are obtained using the maximum likelihood method. The evaluation of the estimators is assessed by conducting a simulation study. Finally, the usefulness and applicability of the new beta power very flexible Weibull distribution are shown by analyzing two engineering data sets. Using four information criteria, it is observed that the new beta power very flexible Weibull distribution is the best-suited model for dealing with failure times data sets.

## 1 Introduction

Capturing the mixed state or complex form of real phenomena is of greater importance to obtain more precise estimates and make accurate decisions. The selection and implementation of a suitable and appropriate probability model for capturing the mixed state behavior of real-life data are very crucial. The selection of an inappropriate probability model to use for analyzing data sets with complex nature often leads to poor and misguided results; see Klakattawi et al. [1]. Therefore, to provide the best description of the real-life data, researchers are working to enhance the distributional flexibility to achieve the highest degree of best fitting; see Bakr et al. [2], Al-Babtain et al. [3], and Jamal et al. [4], among others.

Among the available probability distributions (i.e., proposed, studied, and applied) the two-parameter Weibull model has attracted many researchers for data modeling in applied sectors. Due to its closed-form cumulative distribution function (CDF) and different monotonic hazard function (HF), the Weibull distribution is a very competent probability distribution. For analyzing the biomedical and reliability phenomena, most often the Weibull distribution is the first choice of many researchers to implement. For instance, (i) Liu et al. [5] used a generalized version of the Weibull model for analyzing healthcare events, and (ii) Ghazal and Radwan [6] implemented another modified form of the Weibull model for analyzing the engineering data sets. For a brief review of the interesting modifications of the Weibull distribution with applications in applied sectors; see Almalki and Nadarajah [7].

Suppose *W* be the Weibull distributed random variable with parameters α>0 and σ>0, if its CDF G(w;α,σ) is given by

(1) $$G\left(w;\alpha ,\sigma \right)=1-e^{-\sigma w^{\alpha }},\;w\geq 0.$$

Corresponding to G(w;α,σ) in Eq. (1), the HF, say h(w;α,σ), is expressed by

$$h\left(w;\alpha ,\sigma \right)=\alpha \sigma w^{\alpha -1},\;w>0.$$

For fixed σ=1 and different values of *α*, some visual illustrations of h(w;α,σ) of the Weibull distribution are presented in Fig. 1.

**Figure 1:** Graphical display of h(w;α,σ) of the Weibull distribution for fixed *σ* = 1 and different values of *α*.

From Fig. 1, we can easily observe that the Weibull distribution has three possible shapes of its h(w;α,σ). These shapes include

• Increasing behavior, when α>1 and σ=1,
• Constant behavior, when α=1 and σ=1,
• Decreasing behavior, when α<1 and σ=1.

We can see that Fig. 1 only justifies the monotonic shapes of h(w;α,σ) of the Weibull distribution. However, when the failure behavior (or HF) of the data sets is in a mixed state, the Weibull distribution does not provide the best-suited fit to such kind of complex data sets. To handle this deficiency and increase the ability of the Weibull distribution, a series of new interesting and flexible modifications of the Weibull distribution have been introduced and implemented for modeling the healthcare, reliability, meteorology, sports, and financial scenarios, etc. Some famous and interesting modifications of the Weibull distribution include the (i) flexible Weibull extension; see Bebbington et al. [8], (ii) modified Weibull; see Sarhan and Zaindin [9], (iii) beta-modified Weibull; see Silva et al. [10], (iv) new modified Weibull; see Almalki and Yuan [11], (v) additive modified Weibull; see He et al. [12], and (vi) reduced new modified Weibull; see Almalki [13].

Among the existing modifications of the Weibull model, one of the interesting modified forms of the Weibull distribution is called the very flexible Weibull (VF-Weibull) distribution due to Ahmad and Hussain [14]. The CDF G(w;α,σ) of the VF-Weibull distribution with parameters α>0 and σ>0, is expressed by

(2) $$G\left(w;\alpha ,\sigma \right)=1-e^{-e^{\left(\sigma w-\frac{1}{w^{\alpha }}\right)}},\;w\geq 0,$$

with PDF (probability density function) g(w;α,σ) given by

(3) $$g\left(w;\alpha ,\sigma \right)=\left(\sigma +\frac{\alpha }{w^{\alpha +1}}\right)e^{\left(\sigma w-\frac{1}{w^{\alpha }}\right)}e^{-e^{\left(\sigma w-\frac{1}{w^{\alpha }}\right)}},\;w>0.$$

In this paper, we also introduce a new version of the Weibull distribution for modeling the reliability data sets possessing the mixed state HF. The proposed model is called a new beta power very flexible Weibull (NBPVF-Weibull) distribution. The NBPVF-Weibull is introduced by combining Eq. (2) with the beta power transformation method of Ahmad et al. [15] with CDF F(w;β) given by

(4) $$F\left(w;\beta \right)=\frac{\beta^{G\left(w\right)}-\overset{¯}{G}\left(w\right)}{\beta },\;w\in R,\beta >0,\beta \neq 1,$$

and PDF f(w;β) expressed by

(5) $$f\left(w;\beta \right)=\frac{g\left(w\right)}{\beta }\left[1+\left(\log\beta \right)\beta^{G\left(w\right)}\right],\;w\in R,$$

where $g\left(w\right)=\frac{d}{dw}G\left(w\right)$ and $\overset{¯}{G}\left(w\right)=1-G\left(w\right)$.

In Section 2, we combine Eq. (2) with Eq. (4) and introduce a new probability distribution called a NBPVF-Weibull distribution. Furthermore, the visual description of the PDF and HF of the NBPVF-Weibull is also provided.

## 2 The NBPVF-Weibull: the proposed distribution

Assume W>0 follows the VF-Weibull distribution with CDF G(w;α,σ) given by Eq. (1). Then, for β≠1, the CDF F(w;β,α,σ) and survival function (SF) S(w;β,α,σ) of the NBPVF-Weibull distributed random variable, say *W*, are given by

(6) $$F\left(w;\beta ,\alpha ,\sigma \right)=\frac{\beta^{1-e^{-e^{\left(\sigma w-\frac{1}{w^{\alpha }}\right)}}}-e^{-e^{\left(\sigma w-\frac{1}{w^{\alpha }}\right)}}}{\beta },\;w\geq 0,\beta >0,\beta \neq 1,$$

and

$$S\left(w;\beta ,\alpha ,\sigma \right)=\frac{\beta -\beta^{1-e^{-e^{\left(\sigma w-\frac{1}{w^{\alpha }}\right)}}}+e^{-e^{\left(\sigma w-\frac{1}{w^{\alpha }}\right)}}}{\beta },\;w>0.$$

We can see that for β=1, the CDF F(w;β,α,σ) in Eq. (6) reduces to the CDF G(w;α,σ) of the VF-Weibull distribution presented by Eq. (2).

Using Eq. (2) and Eq. (3) in Eq. (5), we get the PDF f(w;β,α,σ) of the PBPVF-Weibull distributed random variable, given by

(7) $$f\left(w;\beta ,\alpha ,\sigma \right)=\frac{\left(\sigma +\frac{\alpha }{w^{\alpha +1}}\right)e^{\left(\sigma w-\frac{1}{w^{\alpha }}\right)}e^{-e^{\left(\sigma w-\frac{1}{w^{\alpha }}\right)}}}{\beta }\left[1+\left(\log\beta \right)\beta^{1-e^{-e^{\left(\sigma w-\frac{1}{w^{\alpha }}\right)}}}\right],\;w>0.$$

Corresponding to F(w;β,α,σ) and f(w;β,α,σ), the HF h(w;β,α,σ) and cumulative HF H(w;β,α,σ) of the NBPVF-Weibull distribution are given, respectively, by

$$h\left(w;\beta ,\alpha ,\sigma \right)=\frac{\left(\sigma +\frac{\alpha }{w^{\alpha +1}}\right)e^{\left(\sigma w-\frac{1}{w^{\alpha }}\right)}e^{-e^{\left(\sigma w-\frac{1}{w^{\alpha }}\right)}}}{\beta -\beta^{1-e^{-e^{\left(\sigma w-\frac{1}{w^{\alpha }}\right)}}}+e^{-e^{\left(\sigma w-\frac{1}{w^{\alpha }}\right)}}}\left[1+\left(\log\beta \right)\beta^{1-e^{-e^{\left(\sigma w-\frac{1}{w^{\alpha }}\right)}}}\right],\;w>0,$$

and

$$H\left(w;\beta ,\alpha ,\sigma \right)=-\log\left(\frac{\beta -\beta^{1-e^{-e^{\left(\sigma w-\frac{1}{w^{\alpha }}\right)}}}+e^{-e^{\left(\sigma w-\frac{1}{w^{\alpha }}\right)}}}{\beta }\right),\;w>0.$$

For different values of β,α, and *σ*, some visual descriptions of f(w;β,α,σ) of the NBPVF-Weibull distribution are presented in Fig. 2. The plots of f(w;β,α,σ) in Fig. 2, show that f(w;β,α,σ) of the NBPVF-Weibull distribution has different shapes such as bimodal (red curve), uni-modal (green curve), decreasing (blue-curve), and decreasing-increasing-decreasing (gray, magenta, and gold curves).

**Figure 2:** Some visual descriptions of f(w;β,α,σ) of the NBPVF-Weibull distribution including bimodal, uni-modal, and decreasing provided in panels (a-c) and decreasing-increasing-decreasing provided in panel (d).

The plots of h(w;β,α,σ) of the NBPVF-Weibull distribution for different values of β,α, and *σ* are presented in Fig. 3. The plots of h(w;β,α,σ) in Fig. 3, reveal that h(w;β,α,σ) of the NBPVF-Weibull distribution has various shapes such as uni-modal (green curve), decreasing-increasing-decreasing (blue curve), bathtub (gold curve), decreasing (red curve), and modified uni-modal (gray curve).

**Figure 3:** Some visual descriptions of h(w;β,α,σ) of the NBPVF-Weibull distribution including uni-modal, decreasing-increasing-decreasing, bathtub, and decreasing provided in panels (a-d) and modified uni-modal provided in panel (e).

## 3 Estimation and simulation

Here, we proceed with two basic aims. First, it provides the derivation (mathematical expressions) of the maximum likelihood estimators (MLEs) $\left({\overset{ˆ}{\alpha }}_{MLE},{\overset{ˆ}{\sigma }}_{MLE},{\overset{ˆ}{\beta }}_{MLE}\right)$ of the parameters (α,σ,β). Second, it offers a simulation study to evaluate the behaviors of ${\overset{ˆ}{\alpha }}_{MLE},{\overset{ˆ}{\sigma }}_{MLE}$, and ${\overset{ˆ}{\beta }}_{MLE}$ of the NBPVF-Weibull distribution.

### 3.1 Estimation

Assume $W_{1},W_{2},...,W_{n}$ be a set of *n* random samples observed from the PDF f(w;β,α,σ) given by Eq. (7). Then, corresponding to f(w;β,α,σ), the likelihood function (LF), say $\lambda \left(\beta ,\alpha ,\sigma |w_{1},w_{2},...,w_{n}\right)$, is expressed by

(8) $$\lambda \left(\beta ,\alpha ,\sigma |w_{1},w_{2},...,w_{n}\right)=\prod_{i=1}^{n}\frac{\left(\sigma +\frac{\alpha }{w_{i}^{\alpha +1}}\right)e^{\left(\sigma w_{i}-\frac{1}{w_{i}^{\alpha }}\right)}e^{-e^{\left(\sigma w_{i}-\frac{1}{w_{i}^{\alpha }}\right)}}}{\beta }\times \left[1+\left(\log\beta \right)\beta^{1-e^{-e^{\left(\sigma w_{i}-\frac{1}{w_{i}^{\alpha }}\right)}}}\right].$$

Corresponding to $\lambda \left(\beta ,\alpha ,\sigma |w_{1},w_{2},...,w_{n}\right)$ in Eq. (8), the log LF, say λ(β,α,σ), is given by

(9) $$\lambda \left(\beta ,\alpha ,\sigma \right)=\sum_{i=1}^{n}\log\left(\sigma +\frac{\alpha }{w_{i}^{\alpha +1}}\right)+\sum_{i=1}^{n}\left(\sigma w_{i}-\frac{1}{w_{i}^{\alpha }}\right)-\sum_{i=1}^{n}e^{\left(\sigma w_{i}-\frac{1}{w_{i}^{\alpha }}\right)}-n\log\beta +\sum_{i=1}^{n}\log\left[1+\left(\log\beta \right)\beta^{1-e^{-e^{\left(\sigma w_{i}-\frac{1}{w_{i}^{\alpha }}\right)}}}\right].$$

The partial derivatives of λ(β,α,σ) of the NBPVF-Weibull distribution in Eq. (9), are given by

$$\frac{\partial }{\partial \alpha }\lambda \left(\beta ,\alpha ,\sigma \right)=\sum_{i=1}^{n}\frac{\left(w_{i}^{\alpha +1}-\alpha \left(\log w_{i}\right)w_{i}^{\alpha +1}\right)}{\left(\sigma +\frac{\alpha }{w_{i}^{\alpha +1}}\right){\left(w_{i}^{\alpha +1}\right)}^{2}}+\sum_{i=1}^{n}\frac{\left(\log w_{i}\right)}{w_{i}^{\alpha }}-\sum_{i=1}^{n}\frac{\left(\log w_{i}\right)e^{\left(\sigma w_{i}-\frac{1}{w_{i}^{\alpha }}\right)}}{w_{i}^{\alpha }}+\left(\log\beta \right)\sum_{i=1}^{n}\frac{\left(\log w_{i}\right)w_{i}^{-\alpha }e^{\left(\sigma w_{i}-\frac{1}{w_{i}^{\alpha }}\right)}e^{-e^{\left(\sigma w_{i}-\frac{1}{w_{i}^{\alpha }}\right)}}\beta^{1-e^{-e^{\left(\sigma w_{i}-\frac{1}{w_{i}^{\alpha }}\right)}}}}{\left[1+\left(\log\beta \right)\beta^{1-e^{-e^{\left(\sigma w_{i}-\frac{1}{w_{i}^{\alpha }}\right)}}}\right]},$$

$$\frac{\partial }{\partial \sigma }\lambda \left(\beta ,\alpha ,\sigma \right)=\sum_{i=1}^{n}\frac{1}{\left(\sigma +\frac{\alpha }{w_{i}^{\alpha +1}}\right)}+\sum_{i=1}^{n}w_{i}-\sum_{i=1}^{n}w_{i}e^{\left(\sigma w_{i}-\frac{1}{w_{i}^{\alpha }}\right)}+\left(\log\beta \right)\sum_{i=1}^{n}\frac{w_{i}^{\alpha }e^{\left(\sigma w_{i}-\frac{1}{w_{i}^{\alpha }}\right)}e^{-e^{\left(\sigma w_{i}-\frac{1}{w_{i}^{\alpha }}\right)}}\beta^{1-e^{-e^{\left(\sigma w_{i}-\frac{1}{w_{i}^{\alpha }}\right)}}}}{\left[1+\left(\log\beta \right)\beta^{1-e^{-e^{\left(\sigma w_{i}-\frac{1}{w_{i}^{\alpha }}\right)}}}\right]},$$

and

$$\frac{\partial }{\partial \beta }\lambda \left(\beta ,\alpha ,\sigma \right)=-\frac{n}{\beta }+\sum_{i=1}^{n}\frac{\beta^{-e^{-e^{\left(\sigma w_{i}-\frac{1}{w_{i}^{\alpha }}\right)}}}\left[1+\left(\log\beta \right)\left(1-e^{-e^{\left(\sigma w_{i}-\frac{1}{w_{i}^{\alpha }}\right)}}\right)\right]}{\left[1+\left(\log\beta \right)\beta^{1-e^{-e^{\left(\sigma w_{i}-\frac{1}{w_{i}^{\alpha }}\right)}}}\right]}.$$

By solving $\frac{\partial }{\partial \alpha }\lambda \left(\beta ,\alpha ,\sigma \right)=0,\frac{\partial }{\partial \sigma }\lambda \left(\beta ,\alpha ,\sigma \right)=0$, and $\frac{\partial }{\partial \beta }\lambda \left(\beta ,\alpha ,\sigma \right)=0$, we obtain the MLEs ${\overset{ˆ}{\alpha }}_{MLE},{\overset{ˆ}{\sigma }}_{MLE}$, and ${\overset{ˆ}{\beta }}_{MLE}$ of the parameters α,σ, and *β*, respectively.

### 3.2 Simulation

In this subsection, we provide a brief simulation study to evaluate the behaviors of the MLEs $\left({\overset{ˆ}{\alpha }}_{MLE},{\overset{ˆ}{\sigma }}_{MLE},{\overset{ˆ}{\beta }}_{MLE}\right)$ of the NBPVF-Weibull distribution. The evaluation of the MLEs is performed by generating random numbers from the NBPVF-Weibull model with PDF f(w;β,α,σ) using the inverse CDF approach. Thus, using the inverse CDF method, random numbers of sizes, say n=50,100,150,...,1000, are generated from the proposed distribution.

For the NBPVF-Weibull model, the simulation study is carried out for different sets of parameter values of α,σ, and *β*. The selected parameter values are given by α=1.2,σ=1.4,β=0.9, α=0.9,σ=1.0,β=0.6, and α=0.7,σ=1.4,β=1.2.

Two evaluation criteria are selected to see the performances of ${\overset{ˆ}{\alpha }}_{MLE},{\overset{ˆ}{\sigma }}_{MLE}$, and ${\overset{ˆ}{\beta }}_{MLE}$. The selected evaluation criteria are given by

• Bias
  $$Bias\left({\overset{ˆ}{\alpha }}_{MLE}\right)=\frac{1}{1000}\sum_{i=1}^{1000}\left({\overset{ˆ}{\alpha }}_{i}-\alpha \right).$$
• Mean square error (MSE)
  $$MSE\left({\overset{ˆ}{\alpha }}_{MLE}\right)=\frac{1}{1000}\sum_{i=1}^{1000}{\left({\overset{ˆ}{\alpha }}_{i}-\alpha \right)}^{2}.$$

For the NBPVF-Weibull distribution, the simulation studies are conducted using the optim() R-function.

The values of evaluation criteria are also computed for ${\overset{ˆ}{\sigma }}_{MLE}$, and ${\overset{ˆ}{\beta }}_{MLE}$. Corresponding to (i) α=1.2,δ=1.4,β=0.9, (ii) α=0.9,δ=1.0,β=0.6, and (iii) α=0.7,δ=1.4,β=1.2, the simulation results are presented in Table 1, Table 2, and Table 3, respectively. Corresponding to the above three sets of parameters, the visual illustrations of the simulation results are also presented visually in Figure 4, Figure 5, Figure 6.

**Table 1:** Simulation results of the NBPVF-Weibull model for *α* = 0.6,*σ* = 1.3, and *β* = 0.9.

*n*	Parameters	MLEs	Bias	MSEs
	*α*	0.6073293	0.007329280	0.005751738
50	*σ*	1.3503630	0.050363018	0.154431492
	*β*	1.1761524	0.276152432	0.786699690

	*α*	0.6030644	0.003064386	0.002539925
100	*σ*	1.3173980	0.017398003	0.082963706
	*β*	1.0328759	0.132875938	0.284167450

	*α*	0.6016946	0.001694608	0.001685471
150	*σ*	1.3239670	0.023967261	0.063101886
	*β*	1.0043314	0.104331432	0.162774670

	*α*	0.6008674	0.000867411	0.001317299
200	*σ*	1.3063080	0.006307521	0.044048635
	*β*	0.9700574	0.070057362	0.098882060

	*α*	0.5993311	-0.00066893	0.000842609
300	*σ*	1.3123160	0.012315672	0.032546001
	*β*	0.9517367	0.051736693	0.070492680

	*α*	0.6005631	0.000563093	0.000629041
400	*σ*	1.3120390	0.012038667	0.024638390
	*β*	0.9397200	0.039719953	0.044382170

	*α*	0.6001629	0.000162869	0.000482578
500	*σ*	1.3037960	0.003796366	0.017894592
	*β*	0.9246839	0.024683909	0.031154560

	*α*	0.5998807	-0.00011926	0.000382991
600	*σ*	1.3031700	0.003170132	0.013584744
	*β*	0.9169465	0.016946521	0.023636610

	*α*	0.5998857	-0.00011428	0.000375218
700	*σ*	1.2999040	-0.00009557	0.012328788
	*β*	0.9136455	0.013645548	0.020075470

	*α*	0.6001260	0.000125998	0.000303425
800	*σ*	1.2973220	-0.00267750	0.011316002
	*β*	0.9087284	0.008728408	0.019935920

	*α*	0.5994815	-0.00051852	0.000266796
900	*σ*	1.3016520	0.001652290	0.008897177
	*β*	0.9107088	0.010708845	0.014636660

	*α*	0.6002959	0.000295864	0.000248219
1000	*σ*	1.3044180	0.004418171	0.008524169
	*β*	0.9111020	0.011102004	0.013910510

**Table 2:** Simulation results of the NBPVF-Weibull model for *α* = 1.1, *σ* = 0.9, and *β* = 1.3.

*n*	Parameters	MLEs	Bias	MSEs
	*α*	1.1267260	0.026725994	0.02669300
50	*σ*	0.9088228	0.008822774	0.05236809
	*β*	1.6677570	0.367756690	1.47751085

	*α*	1.1043680	0.004367971	0.01155696
100	*σ*	0.9089641	0.008964132	0.02827621
	*β*	1.5443650	0.244365060	0.78850054

	*α*	1.1021560	0.002155780	0.00801806
150	*σ*	0.9014471	0.001447063	0.01781605
	*β*	1.4437970	0.143797220	0.43926691

	*α*	1.1014340	0.001434254	0.00614245
200	*σ*	0.8963391	-0.00366090	0.01516087
	*β*	1.4051920	0.105192140	0.33601575

	*α*	1.1026570	0.002657189	0.00401596
300	*σ*	0.9007262	0.000726193	0.00907103
	*β*	1.3646390	0.064639180	0.17809129

	*α*	1.1036350	0.003635102	0.00318303
400	*σ*	0.9005928	0.000592772	0.00716947
	*β*	1.3504500	0.050450001	0.11508758

	*α*	1.0997940	-0.00020570	0.00234664
500	*σ*	0.9027609	0.002760899	0.00500924
	*β*	1.3446480	0.044648070	0.08826488

	*α*	1.1049920	0.004992180	0.00211825
600	*σ*	0.8979057	-0.00209429	0.00443818
	*β*	1.3236530	0.023652830	0.07432455

	*α*	1.1005940	0.000593666	0.00178615
700	*σ*	0.9011512	0.001151163	0.00373754
	*β*	1.3317520	0.031752420	0.06280585

	*α*	1.1008530	0.000852580	0.00144637
800	*σ*	0.8995760	-0.00042400	0.00335438
	*β*	1.3197400	0.019740290	0.05093062

	*α*	1.1011650	0.001165230	0.00131521
900	*σ*	0.8994400	-0.00056003	0.00323881
	*β*	1.3201920	0.020191740	0.04826828

	*α*	1.1003900	0.000390086	0.00113724
1000	*σ*	0.8990256	-0.00097438	0.00295495
	*β*	1.3202760	0.020275730	0.04498337

**Table 3:** Simulation results of the NBPVF-Weibull model for *α* = 1.0,*σ* = 1.5, and *β* = 1.2.

*n*	Parameters	MLEs	Bias	MSEs
	*α*	1.0067588	0.006758825	0.016278033
50	*σ*	1.5240370	0.024036711	0.153247813
	*β*	1.6560680	0.456067540	1.751950110

	*α*	1.0019035	0.001903537	0.007600183
100	*σ*	1.4903210	-0.00967851	0.091865285
	*β*	1.4377310	0.237730790	0.870881720

	*α*	0.9991745	-0.00082549	0.005490326
150	*σ*	1.4849850	-0.01501536	0.069825205
	*β*	1.3740990	0.174099470	0.629384790

	*α*	0.9950893	-0.00491070	0.003743386
200	*σ*	1.5087690	0.008769447	0.048504032
	*β*	1.3558020	0.155802400	0.361754940

	*α*	1.0001225	0.000122463	0.002359963
300	*σ*	1.4888300	-0.01116952	0.033308849
	*β*	1.2580110	0.058010740	0.200151150

	*α*	0.9988919	-0.00110813	0.001859094
400	*σ*	1.4962260	-0.00377402	0.027250353
	*β*	1.2599340	0.059933670	0.158929670

	*α*	1.0006542	0.000654231	0.001531499
500	*σ*	1.5005020	0.000501666	0.021466249
	*β*	1.2601080	0.060108280	0.120215810

	*α*	0.9992053	-0.00079474	0.001236140
600	*σ*	1.4969530	-0.00304733	0.017834731
	*β*	1.2437960	0.043795950	0.095412900

	*α*	0.9994839	-0.00051613	0.001106130
700	*σ*	1.5021030	0.002103119	0.013152463
	*β*	1.2428280	0.042828480	0.075882730

	*α*	0.9983461	-0.00165390	0.000969061
800	*σ*	1.5007210	0.000721336	0.010377326
	*β*	1.2340450	0.034045300	0.057353050

	*α*	0.9992511	-0.00074894	0.000830333
900	*σ*	1.5020940	0.002094024	0.009545542
	*β*	1.2282970	0.028296760	0.048772420

	*α*	1.0010666	0.001066624	0.000748423
1000	*σ*	1.5009720	0.000971810	0.009173874
	*β*	1.2149280	0.024927690	0.048374600

**Figure 4:** The simulations results of the MLEs (a), biases (b) and MSEs (c) of the NBPVF-Weibull model for *α* = 0.6,*σ* = 1.3, and *β* = 0.9.

**Figure 5:** The simulations results of the MLEs (a), biases (b) and MSEs (c) of the NBPVF-Weibull model for *α* = 1.1,*σ* = 0.9, and *β* = 1.3.

**Figure 6:** The simulations results of the MLEs (a), biases (b) and MSEs (c) of the NBPVF-Weibull model for *α* = 1.0,*σ* = 1.5, and *β* = 1.2.

From Table 1, Table 2, Table 3 (numerical description of the simulation study), and Figure 4, Figure 5, Figure 6 (visual description of the simulation study), we can see that as *n* (size of the samples) increases, the

• MLEs of α,σ, and *β* tend to stable.
• Biases of ${\overset{ˆ}{\alpha }}_{MLE},{\overset{ˆ}{\sigma }}_{MLE}$, and ${\overset{ˆ}{\beta }}_{MLE}$ decreases.
• MSEs of ${\overset{ˆ}{\alpha }}_{MLE},{\overset{ˆ}{\sigma }}_{MLE}$, and ${\overset{ˆ}{\beta }}_{MLE}$ decay to zero.

## 4 Applications of the NBPVF-Weibull

Here, we illustrate the applications of the NBPVF-Weibull to show its importance in engineering and other related sectors. To prove the superior performance of the NBPVF-Weibull distribution, we consider and analyze two engineering applications (i.e., data sets) related to the failure of secondary reactor pumps (Data 1) and failure times of electronic machines (Data 2).

### 4.1 Description of the engineering data sets

The first engineering data set is about the failure time of the secondary reactor pumps occurs; see El-Desouky et al. [16]. The second engineering application is about the failure times (noted per 1000 h) of fifty electronic machines reported by Aryal and Elbatal [17].

Corresponding to the engineering applications, the values of certain key statistics are provided in Table 4. Besides the key statistics in Table 4, some descriptive plots of Data 1 and Data 2 are illustrated, respectively, in Fig. 7 and Fig. 8. Besides, the descriptive plots, the observations of Data 1 and Data 2 are also plotted in Fig. 9.

**Table 4:** Some key statistics of Data 1 and Data 2.

Description	Mean	*Q*_1_	*Q*_2_	*Q*_3_
Data 1	1.578	0.310	0.614	2.041
Data 2	3.343	0.207	1.414	4.498

Description	Median	Variance	Minimum	Maximum
Data 1	0.614	3.727	0.062	6.560
Data 2	1.414	17.484	0.036	15.080

Description	Range	Skewness	Kurtosis	Data size *n*
Data 1	6.498	1.364	3.544	23
Data 2	15.044	1.416	4.084	50

**Figure 7:** Some descriptive plots of Data 1 including histogram (a), kernel density (b), box plot (c), and violin (d).

**Figure 8:** Some descriptive plots of Data 2 including histogram (a), kernel density (b), box plot (c), and violin (d).

**Figure 9:** The visual illustration of the observations of Data 1 and Data 2 are provided in panel (a) and panel (b), respectively.

### 4.2 Competing distributions

Using the considered Data 1 and Data 2, we show the superior performances of the NBPVF-Weibull distribution by comparing its results with other selected rival probability distributions. The selected rival distributions are very competent and known probability models for modeling the engineering data sets. The CDFs of the selected rival models are

• Weibull
  $$G\left(w;\alpha ,\sigma \right)=1-e^{-\sigma w^{\alpha }},\;w\geq 0,\alpha ,\sigma >0.$$
• F-Weibull
  $$G\left(w;\alpha ,\sigma \right)=1-e^{-e^{\left(\sigma w-\frac{\alpha }{w}\right)}},\;w\geq 0,\alpha ,\sigma >0,$$
• EF-Weibull
  $$G\left(w;\alpha ,\sigma ,\gamma \right)={\left(1-e^{-e^{\left(\sigma w-\frac{\alpha }{w}\right)}}\right)}^{\gamma },\;w\geq 0,\alpha ,\sigma ,\gamma >0,$$
• E-Weibull
  $$G\left(w;\alpha ,\sigma ,\gamma \right)={\left(1-e^{-\sigma w^{\alpha }}\right)}^{\gamma },\;w\geq 0,\alpha ,\sigma ,\gamma >0.$$

### 4.3 Selection criteria

In this subsection, we consider certain selection criteria (also called information criteria) to compare the NBPVF-Weibull distribution's fitting power with the above selected rival probability models. These information criteria are used to indicate the best-suited distribution for the engineering data sets discussed above. The numerical results of the information criteria are calculated using the formulas:

• Akaike information criterion (AIC)
  2n−2λ(.).
• Consistent AIC (CAIC)
  $$\frac{2nk}{n-k-1}-2\lambda \left(.\right).$$
• Bayesian information criterion (BIC)
  klog⁡(n)−2λ(.).
• Hannan Quinn information criterion (HQIC)
  2klog⁡[log⁡(n)]−2λ(.).

In the formulas of the above information criteria, the terms *k*, *n*, and λ(.) represent the number of the parameters of the probability distribution, number of observations, and the LLF of the fitted model, respectively. It is worth noting that a competing model, with the smallest/minimum values of the selected information criteria, indicates the best fit.

### 4.4 Analysis of Data 1

Here, we apply the NBPVF-Weibull and other rival probability distributions to the waiting time till the failure of secondary reactor pumps occurs. For this data set, the MLEs ${\overset{ˆ}{\alpha }}_{MLE},{\overset{ˆ}{\sigma }}_{MLE},{\overset{ˆ}{\beta }}_{MLE}$, and ${\overset{ˆ}{\gamma }}_{MLE}$ of fitted distributions are reported in Table 5. To ensure that the MLEs ${\overset{ˆ}{\alpha }}_{MLE},{\overset{ˆ}{\sigma }}_{MLE}$, and ${\overset{ˆ}{\beta }}_{MLE}$ of the NBPVF-Weibull distribution have unique solutions, we obtain the graphical evaluation of the profiles of their LLF; see Fig. 10. The profiles plot of the LLF in Fig. 10, confirm unique solutions of ${\overset{ˆ}{\alpha }}_{MLE},{\overset{ˆ}{\sigma }}_{MLE}$, and ${\overset{ˆ}{\beta }}_{MLE}$ of the NBPVF-Weibull distribution. Furthermore, using Data 1, the information criteria of the NBPVF-Weibull distribution and other rival distributions are provided in Table 6. The results in Table 6 show that for the NBPVF-Weibull distribution, the values of the information criteria are AIC = 50.82057, CAIC = 52.08373, BIC = 54.22705, and HQIC = 51.67729. The second best-suited mode for Data 1 is the F-Weibull distribution with AIC = 64.76717, CAIC = 65.36717, BIC = 67.03815, and HQIC = 65.33831.

**Table 5:** The values of ${\overset{ˆ}{\alpha }}_{MLE},{\overset{ˆ}{\sigma }}_{MLE},{\overset{ˆ}{\beta }}_{MLE}$, and ${\overset{ˆ}{\gamma }}_{MLE}$ for Data 1.

Model	${\overset{ˆ}{\alpha }}_{MLE}$	${\overset{ˆ}{\sigma }}_{MLE}$	${\overset{ˆ}{\beta }}_{MLE}$	${\overset{ˆ}{\gamma }}_{MLE}$
NBPVF-Weibull	0.476600	0.2515386	0.9956156	-
F-Weibull	0.260134	0.2083532	-	-
Weibull	0.805826	0.7694012	-	-
E-Weibull	0.334108	2.6840301	-	7.4702907
EF-Weibull	0.223675	0.2153276	-	1.1702569

**Figure 10:** The profiles plot of the LLF of ${\overset{ˆ}{\alpha }}_{MLE},{\overset{ˆ}{\sigma }}_{MLE}$, and ${\overset{ˆ}{\beta }}_{MLE}$ of the NBPVF-Weibull distribution using Data 1 are provided in panels (a), (b), and (c), respectively.

**Table 6:** The values of the selected criteria of the fitted models for Data 1.

Model	AIC	CAIC	BIC	HQIC
NBPVF-Weibull	50.82057	52.08373	54.22705	51.67729
F-Weibull	64.76717	65.36717	67.03815	65.33831
Weibull	69.02827	69.62827	71.29926	69.59942
E-Weibull	69.68103	70.94419	73.08751	70.53775
EF-Weibull	66.67745	67.94061	70.08393	67.53417

In addition to the numerical evaluation in Table 6, we also compare the NBPVF-Weibull distribution with other distributions through graphical approaches. For the graphical comparison, we obtain the fitted PDF, empirical CDF, Kaplan Meier survival function, and quantile-quantile (QQ) plots; see Fig. 11. The graphical comparison in Fig. 11, reveals the close fit and suitability of the NBPVF-Weibull distribution for analyzing the failure times of the secondary reactor pumps.

**Figure 11:** Using Data 1, the visual illustration of the performances for the NBPVF-Weibull are provided in panels (a-d), for the F-Weibull are provided in panels (e-h), for the Weibull are provided in panels (i-l), for the E-Weibull are provided in panels (m-p), and for the EF-Weibull are provided in panels (q-t).

### 4.5 Analysis of Data 2

Here, we show the second application of the NBPVF-Weibull distribution by considering the failure times of electronic machines (per 1000 h). Using Data 2, we compare the results (using the numerical and visual approaches) of the NBPVF-Weibull distribution with the above rival probability models. Corresponding to Data 2, the values of ${\overset{ˆ}{\alpha }}_{MLE},{\overset{ˆ}{\sigma }}_{MLE},{\overset{ˆ}{\beta }}_{MLE}$, and ${\overset{ˆ}{\gamma }}_{MLE}$ are reported in Table 7. Here, we again confirm the unique solutions of ${\overset{ˆ}{\alpha }}_{MLE},{\overset{ˆ}{\sigma }}_{MLE}$, and ${\overset{ˆ}{\beta }}_{MLE}$ of the NBPVF-Weibull distribution using Data 2. For the second data set, the profiles of the LLF of ${\overset{ˆ}{\alpha }}_{MLE},{\overset{ˆ}{\sigma }}_{MLE}$, and ${\overset{ˆ}{\beta }}_{MLE}$ are plotted in Fig. 12. These plots confirm unique solutions of ${\overset{ˆ}{\alpha }}_{MLE},{\overset{ˆ}{\sigma }}_{MLE}$, and ${\overset{ˆ}{\beta }}_{MLE}$ of the NBPVF-Weibull model. Besides the MLEs, the values of the information criteria are provided in Table 8. Corresponding to the analysis results of Data 2 in Table 8, the NBPVF-Weibull distribution again proves to be the best-suited distribution for considering and analyzing the failure times of electronic machines.

**Table 7:** The values of ${\overset{ˆ}{\alpha }}_{MLE},{\overset{ˆ}{\sigma }}_{MLE},{\overset{ˆ}{\beta }}_{MLE}$, and ${\overset{ˆ}{\gamma }}_{MLE}$ of the fitted models for Data 2.

Model	${\overset{ˆ}{\alpha }}_{MLE}$	${\overset{ˆ}{\sigma }}_{MLE}$	${\overset{ˆ}{\beta }}_{MLE}$	${\overset{ˆ}{\gamma }}_{MLE}$
NBPVF-Weibull	0.415262	0.1105333	1.0736116	-
F-Weibull	0.181734	0.0978508	-	-
Weibull	0.662735	0.5368253	-	-
E-Weibull	0.616219	0.6253129	-	1.1288008
EF-Weibull	0.107669	0.1089219	-	1.7138960

**Figure 12:** The profiles plot of the LLF of ${\overset{ˆ}{\alpha }}_{MLE},{\overset{ˆ}{\sigma }}_{MLE}$, and ${\overset{ˆ}{\beta }}_{MLE}$ of the NBPVF-Weibull distribution using Data 2 are provided in panels (a), (b), and (c), respectively.

**Table 8:** The values of the selected criteria of the fitted models for Data 2.

Model	AIC	CAIC	BIC	HQIC
NBPVF-Weibull	168.4738	168.9955	174.2098	170.6581
F-Weibull	195.8517	196.1070	199.6757	197.3079
Weibull	208.7307	208.9860	212.5547	210.1869
E-Weibull	210.7501	211.2718	216.4862	212.9344
EF-Weibull	193.8878	194.4095	199.6239	196.0721

Besides the numerical comparison in Table 8, we also compare the NBPVF-Weibull distribution with other distributions by using the selected visual comparative tools. For the visual illustration/comparison of the NBPVF-Weibull distribution, we again sketch the plots of the estimated/fitted PDF, empirical CDF, Kaplan Meier survival function, and QQ plots; see Fig. 13. The graphical illustration of the fitting power of the fitted probability distributions shows that the NBPVF-Weibull distribution again performs than the rival probability distributions.

**Figure 13:** Using Data 2, the visual illustration of the performances for the NBPVF-Weibull are provided in panels (a-d), for the F-Weibull are provided in panels (e-h), for the Weibull are provided in panels (i-l), for the E-Weibull are provided in panels (m-p), and for the EF-Weibull are provided in panels (q-t).

## 5 Concluding remarks

In this paper, we studied a novel modified extension of the VF-Weibull distribution by incorporating the beta power transformation method. The proposed modification of the VF-Weibull distribution was called a new beta power very flexible Weibull distribution. The proposed NBPVF-Weibull distribution was able to capture four different shapes of its PDF such as bimodal, decreasing, uni-modal, and decreasing-increasing-decreasing functions. The NBPVF-Weibull distribution was also able to capture five different shapes of its HF such as uni-modal, decreasing-increasing-decreasing, bathtub, decreasing, and modified uni-modal (also called increasing-decreasing-increasing) functions. The MLEs of the NBPVF-Weibull model were mathematically derived and their performances were evaluated through a simulation study. Furthermore, the uniqueness of the MLEs of the NBPVF-Weibull distribution was also shown visually. Finally, two engineering data sets related to the failure times were analyzed to show the superior fitting power of the NBPVF-Weibull distribution. Using certain information criteria, it was shown practically that the NBPVF-Weibull model is the best-suited choice for analyzing the failure times data sets.

## CRediT authorship contribution statement

Faridoon Khan; Ahmad Zubair; Saima K. Khosa; Mohammed Ahmed Alomair; Abdullah Mohammed Alomair; Abdulaziz khalid Alsharidi: Conceived and designed the experiments; Performed the experiments; Analyzed and interpreted the data; Contributed reagents, materials, analysis tools or data; Wrote the paper.

## Declaration of Competing Interest

The authors declare no competing interests.

## Data Availability

Data included in article/supplementary material/referenced in article.
